# Lidocaine inhibits growth, migration and invasion of gastric carcinoma cells by up-regulation of miR-145

**DOI:** 10.1186/s12885-019-5431-9

**Published:** 2019-03-15

**Authors:** Hongyang Sui, Anfeng Lou, Zhisong Li, Jianjun Yang

**Affiliations:** 1 Department of Emergency, The First Affiliated Hospital of Zhengzhou University, Zhengzhou, 450052 China; 2 Department of Anesthesiology, The First Affiliated Hospital of Zhengzhou University, Zhengzhou, 450052 China

**Keywords:** Lidocaine, Gastric cancer, miR-145, MEK/ERK pathway, NF-κB pathway

## Abstract

**Background:**

Gastric cancer receives considerable attention not only because it is the most common cancer all through the world, but also because it’s on the top third leading reason for cancer-related death. Lidocaine is a well-documented local anesthetic that has been reported to suppress cancer development. The study explored the effects of lidocaine on the growth, migration and invasion of the gastric carcinoma cell line MKN45 and the mechanism behind.

**Methods:**

The effect of lidocaine on viability, proliferation and apoptosis of MKN45 cells were analyzed by Cell Counting Kit-8 assay, BrdU staining assay and flow cytometry, respectively. Moreover, cell migration and invasion were both examined by Transwell assay. The expression of apoptosis-, migration-, and invasion-related proteins were detected by western blot. The relative expression of miR-145 was determined by qRT-PCR. Moreover, the impact which lidocaine brought on MEK/ERK and NF-κB pathways were examined by western blot.

**Results:**

Lidocaine inhibited viability, proliferation, migration, and invasion of MKN45 cells, while enhanced apoptosis. Moreover, miR-145 expression was enhanced by lidocaine; and transfection with miR-145 inhibitor increased cell viability, proliferation, migration, and invasion, but inhibited apoptosis. The up-regulation of miR-145 was partly contributed to the inhibitory effect of lidocaine on gastric cancer cell line MKN45. Finally, lidocaine inactivated MEK/ERK and NF-κB pathways via up-regulation of miR-145.

**Conclusions:**

Our results suggested that lidocaine decreased growth, migration and invasion of MKN45 cells via regulating miR-145 expression and further inactivation of MEK/ERK and NF-κB signaling pathways.

## Background

Gastric carcinoma is a catastrophic disease which threats on public health continuingly. Even though the incidence rate in the past years is declined, gastric carcinoma is still standing for over 1,000,000 new cases in 2018 and an approximately 783,000 deaths, which made it to be one of the most common diagnosed cancer with high mortality [1] . Sadly, gastric carcinoma is difficult to be observed in the beginning, but often diagnosed at an advanced stage. The therapeutic strategy with surgical resection combined with chemotherapy or chemoradiation has improved the survival rate of gastric carcinoma patients [2]. However little progress has been made in metastatic gastric cancer and the survival time is only 5 years, which is far away from satisfaction. The sustained attention and research about novel therapeutic options were needed for the treatment of the disease [3].

Lidocaine is a commonly used local anesthetics of amide derivative and a drug to treat ventricular arrhythmia [4]. Lidocaine is used for multiple acute or chronic pain diseases, such as neuropathic pain, inflammatory and nociceptive pains [5, 6]. Recently, lidocaine has been showed to inhibit growth and metastasis in various cancers. For example, lidocaine could inhibit proliferation of bladder cancer BIU-87 cell line in a dose-dependent manner and enhance the actions of some anti-proliferative agents. In tumor-bearing mice, the combination of lidocaine and mitomycin C could prolong survival and reduce bladder wet weight [7]. Lidocaine was showed to significantly increase cell viability and inhibit apoptosis in 5-FU-treated melanoma cells by up-regulating miR-493 [8]. Lidocaine revealed protective effect against breast cancer cells. Lidocaine inhibited migration of breast cancer and also improved survival of mice with peritoneal carcinomatosis [9]. Lidocaine is an effective tumor-inhibitor, but the study about the effect of lidocaine on gastric carcinoma is limited.

miRNAs regulate gene expression by targeting mRNAs and also exert an vital role in modulation of drug efficacy as well as toxicity [10]. Among these identified miRNAs, miR-145 is a common used tumor suppressor in human endometrial cancer [11], non-small cell lung cancer [12], and colorectal cancer [13]. Moreover, miR-145 was found to be down-regulated in gastric cancer [14], which was considered as an important regulator in inhibiting cell growth and development in gastric cancer [15]. Therefore, experiments were performed to investigate the role of miR-145 in gastric cancer cells.

In the current study, the anti-tumor effect of lidocaine in human gastric carcinoma cells MKN45 was studied. Besides, the role of miR-145 in the action of lidocaine was also investigated in order to explore the underlying mechanism. Our findings may provide a new insight for the therapies of gastric carcinoma patients in the future.

## Methods

### Cell culture and treatment

The human gastric cancer cell line MKN45 was provided by Shanghai Institutes for Biological Sciences Cell Resource Center (Shanghai, China) in April of 2016. Before treatment, cells were maintained in liquid nitrogen. The basic information about cell line MKN45 cells were obtained from stomach tissue of 62 years old female patient with gastric cancer. This cell line with adherent phenotype and can be used for transient transfection.

MKN45 cells were maintained in Dulbecco’s modified Eagles medium (DMEM, Gibco, Carlsbad, CA, USA) added with 10% fetal bovine serum (FBS, Gibco, Carlsbad, CA, USA). MKN45 cells were kept in the environment with temperature 37 °C and 5% CO_2_. Lidocaine at different concentrations (1, 5, and 10 mM) was fixed for the cell treatment.

### Cell counting Kit-8 (CCK-8) assay

Cell viability was determined reference to the method used in this lecture [16] . In brief, MKN45 cells were re-plated in 96-well plate (around 5 × 10^3^ cells/well). Then, 10 μl CCK-8 solution (Dojindo Molecular Technologies, Gaithersburg, MD, USA) was added to the DMEM medium. After incubation in the normal atmosphere which made of humidified 95% air with 5% CO_2_ for 1 h.

Cell viability was accessed by determining absorption values (450 nm).

### Proliferation assay

Bromodeoxyuridine (BrdU) is often used to detecting cell proliferation due to its ability in binding to DNA stably. BrdU (Sigma-Aldrich, St. Louis, MO, USA) was added to the MKN45 cells at concentration of 50 μM. Treated cells were counted in more than five visual fields after incubation of 1 h by microscope.

### Apoptosis assay

Cell apoptosis was detected after cells were stained by propidium iodide (PI) and fluorescein isothiocynate (FITC)-conjugated Annexin V. Firstly, MKN45 cells (around 1 × 10^5^ cells/well) were re-plated in 6 well-plate. Then treated cells were washed with cold phosphate buffered saline (PBS) and centrifuged at 2000 rpn for 10 min to resuspend in binding buffer. Then 5 μl Annexin V-FITC was added put in the dark and incubated for 15 min. Similarly, 5 μl PI was added to the plates before analyzed. Finally flow cytometry analysis was carried out using a FACS can (Beckman Coulter, Fullerton, CA, USA).

### Migration and invasion assay

Transwell chamber with the size of pore 8 μm was used for determining cell migratory and invasive abilities. Chamber matrigel invasion 24-well DI kit was provided by BD Biosciences (San Jose, CA) and was used for cell invasion detection. In brief, collected cells from different groups diluted into the density of 1.0 × 10^4^ were administered in in the upper chamber without serum while the lower chamber with complete medium with 10% FBS. Then cells were incubated for 24 h, finally cells in the lower chamber were collected. In the end, collected cells were stained by crystal violet and then counted using a microscope.

### Cell transfection

miR-145 inhibitor and negative control (NC) were transfected into MKN45 cells and then maintained for 24 h. This approach was used to change the expression of miR-145. Cells were diluted into the density of 2 × 10^5^ cells/well and then seeded in new plate and incubated until the cells of 70–80% confluence was reached. MiR-145 inhibitor and the NC were provided by GenePharma Co. (Shanghai, China) and then transfected using Lipofectamine 3000 reagent (Invitrogen, Carlsbad, CA, USA).

### qRT-PCR analysis

Trizol reagent (Life Technologies Corporation, Carlsbad, CA, USA) was used for total RNA extration. Converting miRNA to cDNA was achieved through Taqman MicroRNA Reverse Transcription Kit. In addition, Taqman Universal Master Mix II was used to amplify complementary DNA (cDNA). The TaqMan MicroRNA Assay employ a novel target-specific stem–loop primer during cDNA synthesis to produce a template for real-time PCR to determine the expression of miR-145 (Applied Biosystems, Foster City, CA, USA) The expression of miR-145 was normalized to U6 snRNA.

### Western blot analysis

RIPA lysis buffer (Beyotime, Shanghai, China) supplemented with the protease inhibitors (Roche, Basel, Switzerland) to lysed cells. The equivalent amounts of protein (20 μg) was denatured at 100 °C in loading buffer for 15 min. Afterwards, load samples containing equal amount of proteins and prepared in sample buffer into 8–12% SDS/PAGE wells and transferred to PVDF membranes by voltage gradient transfer. The blots were blocked overnight in 5% nonfat milk. The membranes were incubated with the primary antibodies against Bcl-2 (ab32124), cleaved-Casapse-3 (ab49822), cleaved-Caspase-7 (ab32522), cleaved-Caspase-9 (ab52298), MMP-2 (ab37150), MMP-9 (ab73734), Vimentin (ab8978), MEK (ab32576), p-MEK (ab96379), ERK (ab32537), p-ERK (ab131438), p65 (ab16502), p-p65 (ab86299), IκBα (ab32518), p-IκBα (ab32518), and β-actin (ab8227) purchased from Abcam (Cambridge, UK) at the dilution of 1:1000. Incubate the membrane in primary antibody solutions overnight at 4 °C with gentle rocking. Wash the membrane with 1× TBST three times for 10 min and then incubate the membrane in the appropriate diluted secondary antibody (Abcam). Then the signal was captured and the intensity of the bands was analyzed. Finally result was quantified using Image Lab™ Software (Bio-Rad, Shanghai, China).

### Statistical analysis

All results are manifested as means ± standard deviation (SD) from three to six samples. Data analysis was achieved using Graphpad Prism version 6.0 software (Graph Pad Software, San Diego California, USA). The student *t* test, one-way analysis of variance, and two-way analysis of variance were performed according to the data characteristics. *p* values < 0.05 were treated as significant difference.

## Results

### Lidocaine inhibited growth of MKN45 cells

The MKN45 cell viability, proliferation, and apoptosis were determined after cells were treated by lidocaine. According to CCK-8 assay, cell viability was inhibited after cells were cultured with different concentrations of lidocaine (1, 5 and 10 mM) (Fig. 1a). Due to lidocaine at the concentration of 10 nM and treatment time 48 h, the suppressing effects achieved the most, we chose 10 nM and treatment 48 h in the following experiments. Cell proliferation detected by BrdU was significantly decreased by lidocaine (*p* < 0.01, Fig. 1b). Western blot demonstrated that Cyclin D1 and p21 expression were significantly down-regulated and up-regulated, respectively (*p* < 0.05, Fig. 1c). The apoptotic cell rate was significantly increased by lidocaine (*p* < 0.001, Fig. 1d). Additionally, Western blot data revealed that lidocaine decreased Bcl-2 expression, and increased cleaved-Caspase-3,  -7, and-9 expression (Fig. 1e).

**Fig. 1:** The growth of MKN45 cells was inhibited by lidocaine. Lidocaine (**a**) suppressed cell viability, (**b**) inhibited cell proliferation, (**c**) decreased Cyclin D1 expression and increased p21 expression, (**d**) promoted apoptosis, and (**e**) downregulated Bcl-2 expression, and upregulated cleaved-Caspase-3, -7, and -9 expression. Cell viability, proliferation, apoptosis were detected by Cell Counting kit-8 assay, BrdU assay and flow cytometry, respectively. The accumulated levels of CyclinD1, p21 and apoptotic proteins were analyzed by western blot. *p < 0.05, ** *p* < 0.01, *** *p* < 0.001

### Lidocaine inhibited migration and invasion of MKN45 cells

The MKN45 cell migration and invasion were both analyzed by Transwell assay. Lidocaine inhibited migration (*p* < 0.05, Fig. 2a) and down-regulated MMP-2, and -9 expression (*p* < 0.05, Fig. 2b). In addition, lidocaine inhibited invasion (*p* < 0.001, Fig. 2c) and down-regulated Vimentin expression (*p* < 0.05, Fig. 2d).

**Fig. 2:** The MKN45 cells migration and invasion were inhibited by lidocaine. Lidocaine (**a**) suppressed cell migration, (**b**) reduced MMP-2 and MMP-9 expression, (**c**) suppressed cell invasion, and (**d**) reduced Vimentin expression. Cell migration and invasion were determined by Transwell migration or invasion assay. The accumulated levels of MMP-2, MMP-9 and Vimentin were examined by western blot. *p < 0.05, *** *p* < 0.001

### Lidocaine upregulated the expression of miR-145

Increasing evidence had proved that miR-145 was connected with the gastric cancer [15, 17]. To clarify the mechanism of lidocaine in gastric cancer cells, the relative expression of miR-145 was detected. The data of qRT-PCR revealed that the relative expression of miR-145 was significantly promoted (*p* < 0.01, Fig. 3), which indicated that miR-145 might join in the progression of lidocaine suppressing cell growth.

**Fig. 3:** The relative expression of miR-145 was enhanced by lidocaine treatment. The expression of miR-145 was determined by qRT-PCR. ** *p* < 0.01

### Lidocaine inhibited growth and metastasis of MKN45 cells by up-regulating miR-145

Given that miR-145 has been proposed as a cancer suppressor [18, 19], the role of miR-145 in cancer cell growth, migration and invasion were studied. miR-145 expression was alleviated after transfection with miR-145 inhibitor (*p* < 0.01, Fig. 4a). miR-145 knockdown significantly inhibited the proliferation-inhibitory effect of lidocaine (*p* < 0.01, Fig. 4b). The down-regulation of Cyclin D1 and the up-regulation of p21 were attenuated by miR-145 inhibitor treatment (*p* < 0.001, Fig. 4c). miR-145 knockdown decreased apoptotic cell rate (*p* < 0.001, Fig. 4d), up-regulated Bcl-2 expression, and down-regulated cleaved-Caspase-3, -7, and -9 expression (Fig. 4e). miR-145 knockdown reversed migration-inhibitory effect of lidocaine (*p* < 0.05, Fig. 4f), and increased MMP-2 and MMP-9 expression (*p* < 0.001, Fig. 4g). The down-regulation of miR-145 also significantly increased invasion of MKN45 cells (*p* < 0.01, Fig. 4h) and up-regulated Vimentin expression (*p* < 0.001, Fig. 4i). These data indicated that lidocaine inhibited MKN45 cell growth, migration and invasion through up-regulation of miR-145.

**Fig. 4:** Lidocaine induced inhibition of growth and metastasis of MKN45 cells were attenuated by miR-145 silence. **a** miR-145 expression was decreased after transfection with miR-145 inhibitor. miR-145 knockdown (**b**) increased cell proliferation, (**c**) up-regulated Cyclin D1 expression and down-regulated p21 expression, (**d**) inhibited apoptosis, (**e**) increased Bcl-2 expression, decreased cleaved-Caspase-3, -7, and -9 expression. miR-145 knockdown (**f**) increased migration, (**g**) up-regulated MMP-2 and MMP-9 expression, (**h**) increased invasion, and (**i**) up-regulated Vimentin. *p < 0.05, ** *p* < 0.01, *** *p* < 0.001

### Lidocaine inhibited activations of MEK/ERK and NF-κB pathways by up-regulating miR-145

The underlying mechanism of miR-145 in the function of lidocaine in signal pathways was investigated. Two pathways MEK/ERK and NF-κB were found to be related with the effect of lidocaine and miR-145. Western blot demonstrated that lidocaine significantly alleviated the phosphorylation levels of MEK and ERK (*p* < 0.01, Fig. 5a), as well as the phosphorylation levels of p65 and IκBα (*p* < 0.001, Fig. 5b). However, miR-145 silence exerted the contrary effects on phosphorylation levels of p-MEK, p-ERK, p-p65, and p-IκBα. These data suggested that lidocaine inhibited activations of MEK/ERK and NF-κB pathways possibly by up-regulating miR-145.

**Fig. 5:** Lidocaine inhibited MEK/ERK and NF-κB pathways by up-regulating miR-145. **a** The phosphorylation of MEK/ERK and (**b**) p65 and IκBα were decreased by lidocaine. The phosphorylation of MEK/ERK, p65 and IκBα were analyzed by western blot. ** *p* < 0.01, *** *p* < 0.001

## Discussion

A substantial amount of clinical data demonstrated that anesthetics are still the optimal and most often used method to decrease nociceptive input. Interestingly, the recent evidence has revealed that anesthesia could also affect the progress of the cancer [20]. Lidocaine is a commonly used local anesthetic, which is showed to function in various types of cancers. Our study explored the inhibitory effect of lidocaine on growth, migration and invasion of gastric cancer cell line MKN45. miR-145, an important regulator of gastric cancer [21], is found to be up-regulated by lidocaine. Based on that, we also analyzed the role of miR-145 in the suppressing functions of lidocaine in MKN45 cells.

According to our data, lidocaine significantly inhibited viability, proliferation, migration and invasion of MKN45 cells, but promoted cell apoptosis. The anti-cancer effects of lidocaine were widely reported. Lidocaine inhibited cell invasion and migration of cancer cell lines MDA-MB-231, PC-3 and ES-2 by down-regulation of transient receptor potential cation channel subfamily V member 6 (TRPV6) [22]. Lidocaine decreased the proliferation of lung cancer A549 and H1299 cells by regulating cell cycle in a dose-dependent manner [23]. Lidocaine could also suppress glioma cell growth by blocking TRPM7 channels [24]. All of these previous findings were consistent with our present study.

Our results further showed that lidocaine caused significant reduction in the proliferation, migration, and invasion and significantly increased apoptosis of MKN45 cells via up-regulating miR-145. The role of miR-145 in regulating the effect of lidocaine was supported by our results showing that transfection with miR-145 inhibitor exhibited the contrary effects on MKN45 cells and impaired the inhibitory effects of lidocaine on MKN45 cells with increased proliferation, migration and invasion, and decreased apoptosis. miR-145 was up-regulated after lidocaine treatment and acted as a gastric cancer suppressor gene in our study. This was lined with former researches, which demonstrated that miR-145 expression was lower in tumors relative to matched normal samples and miR-145 overexpression inhibited cell growth and cell metastasis in gastric cancer cells [25]. miR-145 blocked the cell growth and developmet of gastric cancer cells via decreasing Sp1 expression [15]. Many drugs exert effects via expression of some specific genes. Moreover, drug function can be influenced by alternation of these genes [26]. In the present study, miR-145 modulated the inhibitory effects of lidocaine on MKN45 cells.

Further experiments were performed to disclose the mechanism of lidocaine on MKN45 cells. We analyzed the activations of MEK/ERK and NF-κB signaling pathways after lidocaine treatment. It was found that MEK/ERK pathway exerted an crucial role in development of gastric cancer. For example, MEK/ERK pathway was inhibited after the Chinese medicine Tanshinone IIA suppressed gastric carcinoma AGS cells [27]. The previous evidence showed that MEK/ERK pathway was blocked after gastric cancer or cell lines were inhibited [28, 29], which was similar with our data that MEK/ERK pathway was inhibited in lidocaine-treated cells. NF-κB signaling pathway was a well-known tumor-promoting tunnel [30, 31], which was blocked after lidocaine treatment, indicating that lidocaine played the anti-gastric cancer role partly by down-regulating NF-κB pathway.

## Conclusions

Overall, lidocaine was demonstrated to effectively suppress growth, migration and invasion of gastric cancer cells MKN45. miR-145-modulated dysregulation of PI3K/AKT and NF-κB pathways might explain the mechanism of the anti-gastric cancer function of lidocaine in MKN45 cells. Lidocaine could be a potential effective medicine for gastric cancer treatment.

## Abbreviations

BrdU: Bromodeoxyuridine
FITC: fluorescein isothiocynate
NC: negative control
PBS: phosphate buffered saline
PI: propidium iodide
TRPV6: transient receptor potential cation channel subfamily V member 6
